# Impact of Cold Weather on Setup Errors in Radiotherapy

**DOI:** 10.1155/2021/1463299

**Published:** 2021-11-11

**Authors:** Shuxue Zhao, Xianfa Lu, Jiasen Zou, Zhouying Xu, Siyu Wei, Liping Li, Qingguo Fu

**Affiliations:** ^1^Radiotherapy Center, Guangxi Medical University Cancer Hospital, Nanning, Guangxi 530021, China; ^2^Pediatric Department, The First Affiliated Hospital of Guangxi Medical University, Nanning, Guangxi 530021, China

## Abstract

**Objective:**

To investigate the influence of cold weather on setup errors of patients with chest and pelvic disease in radiotherapy.

**Methods:**

The image-guided data of the patients were collected from the Radiotherapy Center of Cancer Hospital Affiliated to Guangxi Medical University from October 2020 to February 2021. During this period, the cold weather days were December 15, 16, and 17, 2020, and January 7 and 8, 2021. For body fixation in radiotherapy, an integrated plate and a thermoplastic mold were employed in 18 patients with chest disease, while an integrated plate and a vacuum pad were applied in 19 patients with pelvic disease. All patients underwent cone beam computed tomography (CBCT) scans in the first five treatments and once a week thereafter. The obtained data were registered to the planning CT image to get the setup errors of the patient in the translational direction including *X*, *Y*, and *Z* axes and rotational direction including *R*_*X*_, *R*_*Y*_, and *R*_*Z*_. Then, the Mann–Whitney *U* test was performed. The expansion boundary values of the chest and pelvis were calculated according to the formula *M*_PTV_=2.5∑+0.7*δ*.

**Results:**

A total of 286 eligible results of CBCT scans were collected. There were 138 chest CBCT scans, including 26 taken in cold weather and 112 in usual weather, and 148 pelvic CBCT scans, including 33 taken in cold weather and 115 in usual weather. The *X*-, *Y*-, and *Z*-axis translational setup errors of patients with chest disease in the cold weather group were 0.16 (0.06, 0.32) cm, 0.25 (0.17, 0.52) cm, and 0.35 (0.21, 0.47) cm, respectively, and those in the usual weather group were 0.14 (0.08, 0.29) cm, 0.23 (0.13, 0.37) cm, and 0.18 (0.1, 0.35) cm, respectively. The results indicated that there was a statistical difference in the *Z*-axis translational error between the cold weather group and the usual weather group (*U* = 935.5; *p*=0.005 < 0.05), while there was no statistical difference in the rotational error between the two groups. The external boundary values of *X*, *Y*, and *Z* axes in the cold weather group were 0.57 cm, 0.92 cm, and 0.99 cm, respectively, and those in the usual weather group were 0.57 cm, 0.78 cm, and 0.68 cm, respectively. There was no significant difference in the translational and rotational errors of patients with pelvic disease between the cold weather group and the usual weather group (*p* < 0.05). The external boundary values of *X*, *Y*, and *Z* axes were 0.63 cm, 0.79 cm, and 0.68 cm in the cold weather group and 0.61 cm, 0.79 cm, and 0.61 cm in the usual weather group, respectively.

**Conclusion:**

The setup error of patients undergoing radiotherapy with their bodies fixed by an integrated plate and a thermoplastic mold was greater in cold weather than in usual weather, especially in the ventrodorsal direction.

## 1. Background

Roentgen first discovered X-ray in 1985 and Madame Curie discovered radium in 1986. After more than a hundred years of development, tumor radiotherapy has become one of the important means to treat malignant tumors. With the progress of science and technology, PET/CT, MRI, and other equipment have promoted the diagnosis of tumors and delineation of target areas to the molecular level. Radiotherapy planning has developed from the past forward planning to reverse planning due to the rapid advances in computer technology. The radiotherapy implementation has developed from two-dimensional radiotherapy to three-dimensional conformal radiotherapy, intensity-modulated radiotherapy, and image-guided radiotherapy due to the development of materials science, engineering, imaging, and so on. The progress indicates that radiotherapy has entered the stage of precise diagnosis, precise planning, and precise implementation. With the arrival of the precise radiotherapy era, the transition in dose distribution between tumor target area and normal tissues and organs needs to be very steep, because of the “win-win or lose-lose” relationship between tumor target area and normal tissues and organs in radiotherapy. There will be no benefit for any side if a tiny miscalculation occurs; thus, higher requirements for the setup in radiotherapy are put forward. Scholars have studied the effects of body weight [1–3], respiration [4–6], body position fixation, molds [7–9], registration mode between planning images and CT images [10–12], and whether to wear a mask during the epidemic of COVID-19 [13–15] on the setup repeatability. To our best knowledge, few studies considered the weather conditions. Therefore, this study aimed to investigate the influence of cold weather on setup errors in radiation therapy.

## 2. Materials and Methods

### 2.1. General Information

The clinical data of patients who underwent image-guided chest and pelvic radiotherapy in our radiotherapy center from October 2020 to February 2021 (December 15, 16, and 17, 2020; January 7 and 8, 2021) were collected. The data obtained on cold weather days (December 15, 16, and17, 2020; January 7 and 8, 2021) and noncold weather days were assigned to the cold weather group and the usual weather group, respectively. There were 18 patients with chest disease, including 14 females and four males. Their ages ranged from 28 to 70 years with a mean age of 51.6 years. There were 19 patients with pelvic disease; they were all females, with an age range from 38 to 78 years and a mean age of 55.9 years. The detailed data are shown in Table 1.

### 2.2. Inclusion Criteria of Setup Error Data

- The included data in the cold weather group should be the CBCT results on cold weather days.
- If the CBCT conducted in cold weather was the first five CBCT examinations of a patient and no setup error correction was ever implemented, all the CBCT data of the patient should be included. If setup error correction was conducted after the fifth time, only the data of the first five CBCT examinations were included.
- If the CBCT conducted in cold weather was not the first five CBCT examinations of a patient and no setup error correction was ever implemented, all the CBCT data of the patient should be included. If the setup error correction was conducted after the fifth time, the data of the first five CBCT examinations were excluded.

### 2.3. Molding and Positioning

Patients with chest disease were laid supine on an integrated plate (Klarity, China). The median sagittal plane of the body was vertical to the bed surface, and the patient's upper limb was bent and lifted in a natural state to the hand support device. The thermoplastic mold (Create, China) that was able to fix the head, neck, and chest was used for fixation, as shown in Figure 1. Patients with pelvic disease were placed in a supine position, and their bodies were fixed with an integrated plate (Klarity, China) and a vacuum pad (Klarity, China). The midline of the body was vertical to the bed surface, and the patient's upper limb was bent and lifted in a natural state to the hand support device, with the toes forward and the feet together, as shown in Figure 2. The positioning of all patients with chest and pelvic disease was performed with a large-aperture dedicated CT simulator (GE LightSpeed™ RT spiral CT) produced by General Motors, USA, using a slice thickness of 5 mm. For patients with chest disease, the positioning mark point was delineated on the thermoplastic mold at the target area position using a pen; for patients with pelvic disease, the positioning mark point was made on the skin at the level of the tumor target area using a laser gun.

### 2.4. Planning and Design

The CT simulated positioning images obtained by planning design were transmitted to the planning system (Philips Pinnacle 9.10) through the DICOM local area network to develop the radiotherapy plan. The target area was delineated regarding the ICRU83 reporting standard. The gross tumor volume (GTV), clinical target volume (CTV), planning tumor volume (PTV), and organ at risk (OAR) were delineated. The physicist completed the design of the plan, and the superior physician and physicist jointly completed the evaluation of the plan. After completion of the radiotherapy treatment plan, it was transmitted to the MOSAIQ system, and the control accelerator (Elekta Synergy System) performed the treatment accordingly.

### 2.5. Image Guidance and Setup Error Data

All validations were performed by two experienced radiotherapists using Elekta X-ray volumetric imaging (XVI) software (version 4.5; Elekta Oncology Systems). Before each treatment, X-ray volumetric images were collected employing isocentric setups through airborne kilovoltage CBCT (XVI 4.5, Elekta Oncology Systems). Scanning parameters were 120 kV, collimator M20, filter F1, scanning angle 0°–180°, and clockwise direction. Each patient had a pretreatment CBCT scan in the first five treatments and weekly treatments thereafter. The treatment plan and planning CT images were transmitted to the XVI system through the network. In the obtained CBCT image, the three-dimensional volume containing the target area was set by selecting the corresponding three-dimensional matching frame. The setting range of the matching frame included the tumor and a few surrounding tissues, avoiding the tissues and organs with great movement changes including the heart as far as possible. Through the match between this three-dimensional volume and the corresponding three-dimensional volume in the planning CT, the three-dimensional setup error could be obtained. CBCT match for the patients with chest disease was performed using grayscale automatic matching and manual registration if necessary. CBCT match for patients with pelvic disease was performed using automatic bone matching and manual registration if necessary, and the setting range of the matching frame included the tumor and its nearby bone structures. The setup error data in cold weather and usual weather were obtained, including the values of left-right direction (*X*), head-foot direction (*Y*), anteroposterior direction (*Z*), rotational coronal position (*R*_*X*_), sagittal position (*R*_*Y*_), and transverse position (*R*_*Z*_). The unit of translational direction was centimeter (cm), and the unit of rotational direction was degree (°). The setup error of each patient was calculated according to the method described by Stroom et al. [16]. All data errors were derived from two aspects: system error and random error. The system error ∑ (represented by the mean value of all setup errors) was mainly derived from the mechanical parameter errors of the simulated positioning machine and the treatment accelerator; the random error *δ* (represented by the standard deviation of all setup errors) was mainly the difference in the repeatability of each setup during radiotherapy [17]. According to VanHerk's [18] study, the calculation formula of CTV to PTV expansion in *X*, *Y*, and *Z* directions was *M*_PTV_=2.5∑+0.7*δ*. The expansion range was calculated accordingly.

### 2.6. Statistical Analysis

Statistical analysis of the data was carried out using SPSS 17.0 statistical software. Since the setup error in all directions did not follow a normal distribution, it was expressed as median (25th percentile, 75th percentile), namely, *M* (*P*25, *P*75). The Mann–Whitney *U* test was employed, and *P* < 0.05 was considered statistically significant.

## 3. Results

### 3.1. General Data

A total of 286 eligible results of CBCT scans were collected. There are 138 chest scans including 26 scans taken in cold weather and 112 in usual weather, and 148 pelvic cavity scans including 33 taken in cold weather and 115 in usual weather.

### 3.2. Comparison of Translational Setup Errors of Patients with Chest Disease in Different Groups

The translational and rotational setup errors of patients with chest disease in different groups are shown in Figure 3. The *X*-, *Y*-, and *Z*-axis translational setup errors of patients with chest disease in the cold weather group were 0.16 (0.06, 0.32) cm, 0.25 (0.17, 0.52) cm, and 0.35 (0.21, 0.47) cm, respectively. The *X*-, *Y*-, and *Z*-axis translational setup errors of patients with chest disease in the usual weather group were 0.14 (0.08, 0.29) cm, 0.23 (0.13, 0.37) cm, and 0.18 (0.1, 0.35) cm, respectively. There was a statistical difference in *Z*-axis translational error between the two groups (*U* = 935.5, *P*=0.005 < 0.05). The *P* values of other directions between the two groups were all greater than 0.05, indicating no significant differences. The detailed data are shown in Table 2.

### 3.3. Comparison of Rotational Setup Errors of Patients with Chest Disease in Different Groups

The *R*_*X*_, *R*_*Y*_, and *R*_*Z*_ rotational setup errors of patients with chest disease in the cold weather group were 0.9 (0.38, 1.73)°, 0.75 (0.4, 1.2)°, and 0.75 (0.35, 1.1)°, respectively. The *R*_*X*_, *R*_*y*_, and *R*_*z*_ rotational setup errors in the usual weather group were 0.8 (0.4, 1.2)°, 0.7 (0.3, 1.4)°, and 0.7 (0.2, 1.1)°, respectively. There were no significant differences in rotational errors between the two groups (*P* > 0.05). The detailed data are shown in Table 3.

### 3.4. Comparison of Translational Setup Errors of Patients with Pelvic Disease in Different Groups

The translational and rotational setup errors of patients with pelvic disease in different groups are shown in Figure 4. The *X*-, *Y*-, and *Z*-axis translational errors of patients with pelvic disease in the cold weather group were 0.17 (0.09, 0.29) cm, 0.21 (0.1, 0.4) cm, and 0.17 (0.07, 0.31) cm, respectively. The *X*-, *Y*-, and *Z*-axis translational errors in the usual weather group were 0.13 (0.06, 0.3) cm, 0.23 (0.11, 0.39) cm, and 0.22 (0.08, 0.32) cm, respectively. There were no significant differences in translational errors between the two groups. The detailed data are shown in Table 4.

### 3.5. Comparison of the Mean Rotational Setup Error of Patients with Pelvic Disease in Different Weather

The mean *R*_*X*_, *R*_*Y*,_ and *R*_*Z*_ rotational setup errors of patients with pelvic disease were 1.1 (0.5, 1.8)°, 0.5 (0.2, 0.8)°, and 0.5 (0.3, 0.9)° in the cold weather group and 0.8 (0.4, 1.55)°, 0.6 (0.25, 1.2)°, and 0.5 (0.2, 1.05)° in the usual weather group, respectively. There were no significant differences in rotational errors between the two groups (*P* > 0.05). The detailed data are shown in Table 5.

### 3.6. Comparison of Expansion Boundary outside the Target Area of Patients with Chest Disease in the Two Groups

The expansion boundary outside the target area of the patients in the cold weather group and usual weather group was *X* (0.57, 0.57) cm, *Y* (0.92, 0.78) cm, and *Z* (0.99, 0.68) cm, respectively, as shown in Table 6.

### 3.7. Comparison of Expansion Boundary outside the Target Area of Patients with Pelvic Disease in the Two Groups

The expansion boundary outside the target area of patients with pelvic disease in the cold weather group and usual weather group was *X* (0.63, 0.61 cm), *Y* (0.79, 0.79) cm, and *Z* (0.68, 0.61) cm, respectively, as shown in Table 7.

## 4. Discussion

Most countries and regions around the world experience the change of seasons. Substances show thermal expansion and contraction due to the change of temperature, so as the human body. Radiation therapy for tumors has entered the era of precision, which can achieve complete coverage of the tumor target area with a high dose according to planning requirements while forming a steep dose drop area around the tumor to reduce the toxicity for normal tissues around the target area. Therefore, if the fixed position of cancer patients is slightly changed during radiotherapy, it will lead to the failure of cancer treatment and the aggravation of normal tissue toxicity. Our research institute is in the south of China, although the temperature is not as low as in the north in winter, the wet and cold weather in the south is more pungent compared with the dry and cold weather in the north. This study mainly investigated the influence of weather on the setup error of cancer patients undergoing radiotherapy, providing a reference for clinical practice and future development of artificial intelligence neural networks.

As illustrated previously, there were no significant differences in *X*- and *Y*-axis translational errors and *R*_*X*_, *R*_*Y*_, and *R*_*Z*_ rotational errors of patients with chest disease between the cold weather group and usual weather group. But the *M* value of the cold weather group was higher than that of the usual weather group. It is worth noting that there was a significant difference in *Z*-axis translational error between the two groups (*U* = 935.5, *P*=0.005 < 0.05), which may result from the integrated plate + thermoplastic mold used for the fixation. When the patient takes off the upper body clothes and lay on the plate in cold weather, the contraction of the whole back muscle may be caused by the contraction of the capillaries on the back, which may change the human body thickness in the ventrodorsal direction, resulting in the increase of *Z*-axis error in the registration with the planning image.

There were no significant differences in both translational and rotational setup errors of patients with pelvic disease, which may be because of the vacuum pad used for body fixation in radiotherapy. In cold weather, patients did not feel uncomfortable lying on the pad after undressing. However, the data showed that the *R*_*X*_ value in the cold weather group (2.5°) was higher than that in the usual weather group (2°). A previous study has demonstrated that the rotation angle >2° influences the distribution of planning dose [19]. Therefore, if the setup error angle was great than 2°, it was necessary to reset the position since our linear accelerator was not equipped with a six-dimensional treatment table. The reason for the greater *R*_*X*_ value in the cold weather group might be because the head pad pillow and the vacuum pad wrapped the chest, abdomen, and most of the thighs, while the lower leg and foot are not wrapped in the vacuum pad, which will directly contact the carbon fiber plate of the treatment bed. This made the patient uncomfortable and caused their legs to extend and contract, leading to the increased *R*_*X*_.

As for the M_PTV_ value of CTV to PTV expansion, the external boundary values of *X*, *Y*, and *Z* were 0.57 cm, 0.92 cm, and 0.99 cm in the cold weather group and 0.57 cm, 0.78 cm, and 0.68 cm in usual weather group, respectively. The expansion boundary values in the left and right directions are almost equal. But the values in the head-foot direction and ventrodorsal direction in the cold weather group were 0.14 cm and 0.31 cm larger than that in the usual weather group, respectively. Shen et al. [20] designed a new breast vacuum bag to obtain the *M*_PTV_ boundary values of 0.44 cm, 0.31 cm, and 0.38 cm required for *X*, Y, and *Z*, respectively, which were smaller than those obtained in this study. Deseyne et al. [21] used a modified prone breastplate to obtain the *M*_PTV_ boundary values of 1.14 cm, 1.21 cm, and 1.0 cm required for *X*, *Y*, and *Z*, respectively, which were greater than those obtained in this study. Cravo Sá A et al. [22] employed 3D surface image guidance to achieve the expanded *M*_PTV_ boundary values of 0.89 cm, 10.4 cm, and 0.93 cm required for *X*, *Y*, and *Z*, respectively, which were greater than the values in the usual weather group and similar to those in the cold weather group in this study.

As for the *M*_PTV_ value of CTV to PTV of patients with pelvic disease, the external boundary values of *X*, *Y*, and *Z* were 0.63 cm, 0.79 cm, and 0.68 cm in the cold weather group and 0.61 cm, 0.79 cm, and 0.61 cm in the usual weather group, respectively. They were almost equal. Singh et al. [23] applied EPID image guidance to achieve the PTV boundary values required for *X*, *Y*, and *Z*, which were 0.9 cm, 1.0 cm, and 0.6 cm, respectively, when the alignment marker points were added without body fixation. Compared with the values in this study, *X* and *Y* values were larger, while *Z* value was the same. Wu et al. [1] used CBCT image-guided equipment, the *M*_PTV_ boundary values required for *X*, *Y*, and *Z* were 0.40 cm, 0.81 cm, and 0.45 cm, respectively. Compared with the values in this study, the expansion boundary values of *X* and *Z* were smaller, while the expansion boundary value of *Y*-axis was almost the same. Patni et al. [24] employed the CBCT image-guided equipment to achieve the MPTV boundary values required for *X*, *Y*, and *Z*, which were 0.56 cm, 1.03 cm, and 0.58 cm, respectively. The expansion boundary values of *X* and *Z* were smaller, while that of *Y*-axis was larger compared with those in this study. In addition, the largest expansion boundary value was found in *Y*-axis among the three axes in the translational direction, as reported in other studies.

## 5. Conclusion

In conclusion, the setup error of patients treated with radiotherapy in cold weather using the integrated plate and thermoplastic mold fixation will be greater than that in usual weather, especially in the ventrodorsal direction. Therefore, attention must be paid to the possibility of this error in cold weather. The measures that should be taken are as follows. (i) The patient should be asked to arrive at the radiotherapy area about an hour in advance to avoid direct entry to the machine room for treatment. (ii) The air conditioning temperature in the radiotherapy machine room and radiotherapy waiting area can be appropriately increased to ensure the normal operation of radiotherapy equipment. (iii) The integrated plate can be heated to make the patient comfortable when touching it. (iv) In cold weather, the number of image guidance can be increased. (v) For patients with pelvic tumors who need the integrated plate and vacuum pad for fixation in radiotherapy, a large error in the rotation direction (*R*_*X*_) may occur because the heel and lower leg are directly exposed to the ice-cold carbon brazing treatment bed surface. Thus, attention should be paid. A warming soft pad can be laid during positioning and treatment to improve comfort and reduce their movement.

## Figures and Tables

**Figure 1:** Position for patients with thoracic malignancies.

**Figure 2:** Position for patients with pelvic tumors.

**Figure 3:** The translational and rotational setup errors of patients with chest disease.

**Figure 4:** The translational and rotational setup errors of patients with pelvic disease.

**Table 1:** The collected data of the patients.

	Patients with chest disease	Patients with pelvic disease
Number of patients	18	19
Age	51.6 (28–70)	55.9 (38–79)
Gender	Male: 4	Male: 0
	Female: 14	Female: 19
Tumor type	Breast cancer: 14	Uterine cancer: 7
	Esophageal cancer: 2	Cervical cancer: 12
	Lung cancer: 2	
Fixation mode	Integrated plate + thermoplastic mold	Integrated plate + vacuum pad
Number of CBCT	138	148

**Table 2:** Comparison of translational errors between the two groups.

Group	Number of CBCT	Translational errors		
		*X*	*Y*	*Z*
Cold weather group	26	0.16 (0.06, 0.32)	0.25 (0.17, 0.52)	0.35 (0.21, 0.47)
Usual weather group	112	0.14 (0.08, 0.29)	0.23 (0.13, 0.37)	0.18 (0.1, 0.35)
U		1444.5	1264	935.5
*P*		0.95	0.296	0.005

There was a significant difference in *Z*-axis translational error between the two groups (*P* < 0.05).

**Table 3:** Comparison of rotational errors between the two groups.

Group	*n*	Rotational errors		
		*R*_*X*_	*R*_*Y*_	*R*_*z*_
Cold weather group	26	0.9 (0.38, 1.73)	0.75 (0.4, 1.2)	0.75 (0.35, 1.1)
Usual weather group	112	0.8 (0.4, 1.2)	0.7 (0.3, 1.4)	0.7 (0.2, 1.1)
*U*		1378	1413	1357
*P*		0.671	0.815	0.589

There were no significant differences in rotational error between the two groups (*P* > 0.05).

**Table 4:** Comparison of translational errors between the two groups.

Group	Number of CBCT	Translational errors		
		*X*	*Y*	*Z*
Cold weather group	33	0.17 (0.09, 0.29)	0.21 (0.10, 0.40)	0.17 (0.07, 0.31)
Usual weather group	115	0.13 (0.06, 0.3)	0.23 (0.11, 0.39)	0.22 (0.08, 0.32)
*t*		1732.5	1769.5	1701.5
*P*		0.447	0.555	0.366

There was no significant difference in *X*, Y, and *Z* translational errors between the two groups (*P* > 0.05).

**Table 5:** Comparison of rotational errors between the two groups.

Group	Number of CBCT	Rotational errors		
		*R*_*X*_	*R*_*Y*_	*R*_*Z*_
Cold weather group	33	1.1 (0.5, 1.8)	0.5 (0.20, 0.80)	0.5 (0.3, 0.9)
Usual weather group	115	0.8 (0.4, 1.55)	0.6 (0.25, 1.2)	0.5 (0.2, 1.05)
*t*		1607	1700.5	1853
*P*		0.18	0.363	0.837

There was no significant difference in *R*_*X*_, *R*_*Y*_, and *R*_*Z*_ rotational errors between the two groups (*P* > 0.05).

**Table 6:** *M*_PTV_ of CTV to PTV expansion boundary of patients with chest disease in different groups.

Group	*n*	∑			*δ*			*M*_PTV_		
		*X*	*Y*	*Z*	*X*	Y	*Z*	*X*	*Y*	*Z*
Cold weather group	26	0.19	0.31	0.35	0.15	0.21	0.18	0.57	0.92	0.99
Usual weather group	112	0.15	0.21	0.18	0.19	0.26	0.23	0.57	0.78	0.68

**Table 7:** *M*_PTV_ of CTV to PTV expansion boundary of patients with pelvic disease in different groups.

Group	Number of CBCT	∑			*δ*			*M*PTV		
		*X*	*Y*	*Z*	*X*	*Y*	*Z*	*X*	*Y*	*Z*
Cold weather group	33	0.20	0.27	0.23	0.18	0.18	0.16	0.63	0.79	0.68
Usual weather group	115	0.18	0.18	0.16	0.20	0.26	0.20	0.61	0.79	0.61

## Data Availability

The simulation experimental data used to support the findings of this study are available from the corresponding author upon request.
